The article "Isolation and characterization of equine endometrial mesenchymal stromal cells" was published in 2017. Journal: Stem Cell Res Ther.

# Isolation and characterization of equine endometrial mesenchymal stromal cells

**DOI:** 10.1186/s13287-017-0616-0

**Published:** 2017-07-12

**Authors:** B. Elisabeth Rink, Karin R. Amilon, Cristina L. Esteves, Hilari M. French, Elaine Watson, Christine Aurich, F. Xavier Donadeu

**Affiliations:** 1 Ross University School of Veterinary Medicine, Basseterre, Saint Kitts and Nevis; 2 The Roslin Institute, University of Edinburgh, Edinburgh, EH25 9RG UK; 3 University of Veterinary Medicine, 1220 Vienna, Austria; 4 The Roslin Institute, University of Edinburgh, Easter Bush, Midlothian, EH25 9RG UK

**Keywords:** Mesenchymal stem cells, Endometrium, Equine, Horse

## Abstract

**Background:**

Equine mesenchymal stromal/stem cells (MSCs) are most commonly harvested from bone marrow (BM) or adipose tissue, requiring the use of surgical procedures. By contrast, the uterus can be accessed nonsurgically, and may provide a more readily available cell source. While human endometrium is known to harbor mesenchymal precursor cells, MSCs have not been identified in equine endometrium. This study reports the isolation, culture, and characterization of MSCs from equine endometrium.

**Methods:**

The presence of MSC and pericyte markers in endometrial sections was determined using immunohistochemistry. Stromal cells were harvested and cultured after separation of epithelial cells from endometrial fragments using Mucin-1-bound beads. For comparison, MSCs were also harvested from BM. The expression of surface markers in endometrial and BM-derived MSCs was characterized using flow cytometry and quantitative polymerase chain reaction. MSCs were differentiated in vitro into adipogenic, chondrogenic, osteogenic, and smooth muscle lineages.

**Results:**

Typical markers of MSCs (CD29, CD44, CD90, and CD105) and pericytes (NG2 and CD146) were localized in the equine endometrium. Both endometrial and BM MSCs grew clonally and robustly expressed MSC and pericyte markers in culture while showing greatly reduced or negligible expression of hematopoietic markers (CD45, CD34) and MHC-II. Additionally, both endometrial and BM MSCs differentiated into adipogenic, osteogenic, and chondrogenic lineages in vitro, and endometrial MSCs had a distinct ability to undergo smooth muscle differentiation.

**Conclusions:**

We have demonstrated for the first time the presence of cells in equine endometrium that fulfill the definition of MSCs. The equine endometrium may provide an alternative, easily accessible source of MSCs, not only for therapeutic regeneration of the uterus, but also for other tissues where MSCs from other sources are currently being used therapeutically.

## Background

Considerable progress has been made in understanding the biology and therapeutic potential of adult stem cells since the first report of human hematopoietic stem cell transplantation in 1957 [1]. Mesenchymal stem or stromal cells (MSCs) were originally described in the 1960s as a subset of fibroblast-like cells in the bone marrow capable of undergoing osteogenic differentiation [2]. Minimum criteria defining human MSCs were established by the International Society for Cellular Therapy in 2006 [3] and include: plastic adherence under standard culture conditions; expression of the surface markers CD73, CD90, and CD105 and lack of expression of hematopoietic markers as well as HLA-DR; and ability to undergo adipogenic, chondrogenic, and osteogenic differentiation in vitro. In 2013, CD29 and CD44 were added to the list of MSC-positive surface markers [4]. Furthermore, the origin of MSCs in multiple body tissues, including human endometrium [5, 6], has been traced to perivascular cells expressing CD146, NG2, PDGFRβ, and α-SMA. Expression of these markers is maintained by human MSCs in culture [7]. Moreover, studies in vitro and using cell transplantation in model species have shown that, in addition to providing different types of precursor cells, MSCs contribute to tissue repair through immunomodulatory, antiapoptotic, antimicrobial, and a variety of other trophic effects that act to enhance endogenous repair mechanisms [8]. Based on these findings, several hundred clinical trials are currently being carried out using human MSCs [9].

The article "Isolation and characterization of equine endometrial mesenchymal stromal cells" was published in 2017. Journal: Stem Cell Res Ther.

In the horse, MSCs have been used clinically for about 15 years, with therapeutic benefit reported in the treatment of several orthopedic conditions. Equine MSCs are commonly harvested from bone marrow or adipose tissue and are expanded in vitro before use in autologous transplants [10–13]. The requirement to use surgical procedures to harvest cells from those locations has driven the search for other—less invasive—sources including whole blood, umbilical cord blood, or Wharton jelly [14–17]. In that regard, the endometrium represents an attractive alternative source of MSCs in the horse.

Endometrial cells meeting the criteria of MSCs have already been harvested and characterized from humans, rodents, pigs, dogs, and sheep [18–25]. In addition to undergoing trilineage differentiation, they can reportedly generate muscle and neuronal lineages [5, 26]. The therapeutic potential of endometrial MSCs has already been demonstrated in relation to premature ovarian failure [27], Parkinson’s disease [26], and pelvic organ prolapse [28], although these uses have yet to be proven clinically.

The equine endometrium is highly dynamic, cyclically undergoing remodeling [29] which suggests the presence of an active population of mesenchymal precursor cells, yet this has not been investigated. With the goal of eventually exploring the therapeutic potential of these cells, this study aimed to isolate and characterize equine endometrial MSCs and compare their properties to those of the well-characterized bone marrow (BM)-derived MSCs.

The article "Isolation and characterization of equine endometrial mesenchymal stromal cells" was published in 2017. Journal: Stem Cell Res Ther.

## Methods

### Samples and materials

Equine reproductive tracts were collected post mortem from five prepubertal (18-month-old) Welsh Cob ponies and one 6-year-old warmblood mare during diestrus. Bone marrow samples were collected from three Welsh Cob ponies. The animals were euthanized at the School of Veterinary Studies of the University of Edinburgh or the School of Veterinary Medicine of the University of Glasgow for reasons not related to any reproductive tract pathology. All animal procedures were carried out according to the UK Home Office Animals (Scientific Procedures) Act 1986 with approval by the Ethical Review Committee, University of Edinburgh (60/4207). All chemicals and reagents used for cell culture in the study were obtained from Life Technologies (Thermo Fisher Scientific, Paisley, UK) unless otherwise specified, and culture plastic ware (Nunc™) was purchased from Sigma Aldrich (St Louis, MO, USA).

### Immunohistochemistry

Small pieces of equine endometrium (5 mm × 5 mm) were snap frozen and cut into 5-μm sections using a Leica CM1900 cryotome. The tissue sections were fixed in ice-cold methanol:acetone (50:50) for 10 minutes and washed three times with phosphate buffered saline (PBS) before incubation with a Protein Block (Spring Bioscience) for 45 minutes at room temperature. The sections were then incubated overnight at 4 °C with the primary antibodies presented in Table 1. Another three washes with PBS were followed by incubation with the secondary antibody (Table 1) for 30 minutes at room temperature. Finally, the nuclei were counterstained for 3 minutes with 4′,6-diamidine-2′-phenylindole dihydrochloride (DAPI) before mounting. Sections were visualized under a Leica DM LB2 fluorescence microscope.

**Table 1:** Antibodies selected for immunohistochemistry and flow cytometry characterization of equine MSCs

Antibody	Host, isotype	Epitope	Clone	Company
CD29	Mouse, IgG1,κ	Human	TS2/16	BioLegend
CD44	Mouse, IgG1	Horse	CVS18	AbD Serotec
CD90	Mouse, IgG1,κ	Rat	OX-7	BD Pharmingen
CD105	Mouse, IgG1	Human	SN6	AbD Serotec
NG2:APC	Mouse, IgG1	Human	LHM-2	R&D Systems
CD146:FITC	Mouse, IgG1	Human	OJ79c	AbD Serotec
CD34:PE	Mouse, IgG1	Human	4H11[APG]	Immuno Tools
MHC-II:FITC	Mouse, IgG1	Horse	CVS20	AbD Serotec
Mucin-1	Goat, IgG		Polyclonal	Santa Cruz
Secondary antibodies				
IgG—AF568	Donkey	Mouse	Polyclonal	Invitrogen
IgG—AF488	Goat	Mouse	Polyclonal	Invitrogen
IgG—AF568	Donkey	Goat	Polyclonal	Invitrogen
Isotype controls				
Mouse IgG1, κ			MOPC-21	BioLegend
Mouse IgG1			11711	R&D Systems
Mouse IgG1:APC			11711	R&D Systems
Mouse IgG1:PE			PPV-06	Immuno Tools
Mouse IgG1:FITC				AbD Serotec
Goat IgG				Santa Cruz

*MSC* mesenchymal stromal/stem cell

The article "Isolation and characterization of equine endometrial mesenchymal stromal cells" was published in 2017. Journal: Stem Cell Res Ther.

### Isolation of equine endometrial stromal cells

One gram of endometrial tissue was stripped from the underlying myometrium and dissociated using mechanical and enzymatic digestion as described previously [20] with a few modifications. In short, the tissue pieces were washed twice in PBS and minced before dissociation in DMEM/F-12 containing 0.1% bovine serum albumin (BSA), 0.5% collagenase I, 40 μg/ml deoxyribonuclease type I (Sigma Aldrich), and 1% penicillin/streptomycin for 40 minutes at 37 °C in a SI50 Orbital Incubator (Stuart Scientific). The resulting cell solution was filtered through a sterile 70-μm cell strainer (Fisher Scientific) to separate single cells from undigested tissue fragments. After washing with MSC culture medium consisting of DMEM/F-12 containing 10% fetal bovine serum (FBS) and 1% penicillin/streptomycin, and centrifugation for 5 minutes at 720 × *g*, the resulting cell pellet was resuspended in Ca^2+^ and Mg^2+^-free PBS supplemented with 0.1% FBS and 2 mM sodium citrate.

Magnetic Dynabeads M-450 that had been coated with a Mucin-1 antibody (Santa Cruz) according to the manufacturer’s protocol were utilized to remove epithelial cells from the single cell suspension. The number of Mucin-1-coated beads required was calculated assuming 50% of the cell suspension was epithelial. Four beads were incubated per epithelial cell for 40 minutes at 4 °C with gentle rotation and tilting. Unbound (stromal, Muc-1^–^) and bound (epithelial, Muc-1^+^) cell fractions were collected using a Dynamagnet 2, centrifuged, and cultured in MSC culture medium at an initial density of 10^6^ cells/75 cm^2^ in a humidified incubator at 37 °C in 5%CO_2_:95% air. Medium was changed every 2–3 days.

### Isolation of equine bone marrow-derived MSCs

Bone marrow was scraped out of the sternum and immersed in 30 ml PBS containing 45 mg ethylenediaminetetraacetic acid (EDTA) in a 50-ml Falcon tube. The tube was gently rotated and tilted to wash out cells from the bone marrow matrix. The solution was filtered through a 40-μm cell strainer (Fisher Scientific) and centrifuged at 720 × *g* for 5 minutes. The resulting cell pellet was resuspended in PBS. To remove red blood cells, 4 ml of the BM cell solution was underlaid with 3 ml Ficoll Paque PLUS (GE Healthcare) and centrifuged at 20 °C for 40 minutes at 400 × *g*. The interphase layer of mononuclear cells was collected, washed twice with PBS, and cultured at an initial density of 20–40 million cells/175 cm^2^ in MSC culture medium under the same conditions already described for the endometrial-derived stromal cells.

The article "Isolation and characterization of equine endometrial mesenchymal stromal cells" was published in 2017. Journal: Stem Cell Res Ther.

### Colony forming unit assay

Doubling times (DTs) of endometrial Muc-1^–^ fraction cells (*n* = 6 horses) and BM MSCs (*n* = 3 horses) in culture were calculated between passages 1 and 2 using the following equation:

$$ \mathrm{D}\mathrm{T} = T\ { \ln}_2/ \ln \left({X}_{\mathrm{e}}/{X}_{\mathrm{b}}\right), $$

where *T* is the incubation time in days, and *X*_b_ and *X*_e_ are the cell numbers at the beginning and the end, respectively, of the incubation time.

Endometrial Muc-1^–^ fraction cells and BM MSCs, both at passage 2, were seeded in triplicate at clonal densities of 5 and 10 cells/cm^2^ in six-well plates and cultured in MSC medium in a humidified atmosphere at 37 °C in 5% CO_2_:95% air. Medium was changed every 3–4 days, and on the 12th day of culture cells were washed with PBS and fixed with 10% buffered formalin for 1 hour. Cultures were then stained with crystal violet (Sigma Aldrich) for 10 minutes, washed three times with dH_2_O, and dried at room temperature.

Cell clusters that were visible without magnification and contained more than 50 cells were defined as colonies. Cloning efficiency (CE) was calculated with the following formula:

$$ C E=\frac{number\  of\  colonies}{number\  of\  cells\  seeded} \cdot 100 $$

### Flow cytometry

Endometrial Muc-1^–^ cells (*n* = 6 horses) and BM MSCs (*n* = 3 horses) at passage 3 or 4 were analyzed using flow cytometry. The cultured cells were lifted with TrypLE, washed with complete MSC culture medium, and centrifuged at 720 × *g* for 5 minutes at room temperature. Cell pellets were resuspended in PBS containing 5% FBS and incubated for 45 minutes on ice. Cells were then incubated with directly conjugated or unconjugated primary antibodies to different cell surface markers or with matched isotype control IgG (Table 1) for 1 hour at 4 °C. After three washes with PBS, cells were incubated with AF488-conjugated secondary antibodies for 30 minutes at 4 °C. Cells were analyzed using a LSR Fortessa™ flow cytometer (BD Biosciences) equipped with FACS Diva software and the collected data (10000 events) were analyzed with FlowJo (V10; LLC).

Cross-reactivity of cell surface marker antibodies was tested by IHC and flow cytometry, and the expression of each marker was confirmed via RT quantitative polymerase chain reaction (qPCR).

### qPCR analyses

RNA was extracted using TRIzol reagent from freshly collected endometrial cells (*n* = 6 horses) and from cultures of endometrial Muc-1^–^ cells (*n* = 6 horses) and BM MSCs (*n* = 3 horses) at passages 1 and 4. RNA was analyzed using a spectrophotometer (ND-1000, Nano Drop®) and total RNA (0.5–1 μg) was reverse-transcribed using SuperScript III following the instructions of the manufacturer. Subsequent qPCR reactions were performed using SensiFAST™ SYBR® Lo-ROX Kit (Bioline) and equine primers (Table 2) in a Stratagene Mx3000P qPCR machine (Agilent technologies). Data were analyzed with MxPRO qPCR software (Agilent technologies). Values were calculated relative to a standard curve prepared from a pool of samples run simultaneously. Three reference genes were analyzed for stability using the web-based comprehensive tool RefFinder [30] integrating geNorm, BestKeeper, Normfinder, and the comparative ΔCt method. Data were normalized using RNA levels of 18S.

The article "Isolation and characterization of equine endometrial mesenchymal stromal cells" was published in 2017. Journal: Stem Cell Res Ther.

**Table 2:** Primers used for qPCR analysis

Marker		Primer sequence (5′–3′)	
Reference gene	*18S*	Forward	GCT GGC ACC AGA CTT G
		Reverse	GGG GAA TCA GGG TTC G
	*TBP*	Forward	CCA AGC GTT TTG CTG TA
		Reverse	TTC ACT CTT GGC TCC CG
	*GAPDH*	Forward	GAA GAT GTG GCG CGA TGG CC
		Reverse	ACT GAC ACG TTA GGG GTG GGG AC
MSC marker	CD29	Forward	GGC TAA CAG GGA GTT TCA GAT
		Reverse	ACA TCT ATT TTC ATC TGC TTG GC
	CD44	Forward	CCC ACG GAT CTG AAA CAA GTG
		Reverse	TTC TGG AAT TTG AGG TCT CCG TAT
	CD90	Forward	TGC GAA CTC CGC CTC TCT
		Reverse	GCT TAT GCC CTC GCA CTT G
	CD105	Forward	GAC GGA AAA TGT GGT CAG TAA TGA
		Reverse	GCG AGA GGC TCT CCG TGT T
Perivascular marker	CD146	Forward	CTG GAC TTG GAA ACC ACA ACA TC
		Reverse	CAG GTC TCA CTC GGA CAT CAG A
	NG2	Forward	CGA ATC ATT GGG CCC TAC TT
		Reverse	GCT GTT CCA CCT CTC TCC AG
Hematopoietic marker	CD34	Forward	CAC TAA ACC CTC TAC ATC ATT TTC TCC TA
		Reverse	GGC AGA TAC CTT GAG TCA ATT TCA
	CD45	Forward	TGA TTC CCA GAA ATG ACC ATG TA
		Reverse	ACA TTT TGG GCT TGT CCT GTA AC
Epithelial marker	Mucin-1	Forward	CTA TCT CGT TGC CCT GGC TG
		Reverse	GTA GGC ATC ACG GGT TGG AA
Smooth muscle marker	ACTA2	Forward	CTA ACA ACG TCC TCT CCG GG
		Reverse	CTG CTG GAA GGT GGA CAG AG
	CNN1	Forward	CGG CAA CTT CAT GGA CG
		Reverse	TTC TCC AGC TGG TGC CAA T
	MHY11	Forward	ATC CAT CCT GAC CCC ACG TA
		Reverse	CGG AAG AGC CGC TCA TAA GT

*MSC* mesenchymal stromal/stem cell, *qPCR* quantitative polymerase chain reaction

### In-vitro trilineage differentiation

Endometrial Muc-1^–^ cells and BM MSCs (from three horses each) were used separately at passage 3 or 4. For adipogenic differentiation, cells were seeded in triplicate wells of 12-well plates (5000/cm^2^) with MSC culture medium for 2–4 days before changing medium to DMEM/F-12 containing 7% rabbit serum, 3% FBS, 1% penicillin/streptomycin, 1 μM dexamethasone (Sigma Aldrich), 0.5 mM 3-isobutyl-1-methylxanthine (IBMX) (Sigma Aldrich), 10 μg/ml insulin (Sigma Aldrich), and 100 μM indomethacin (Sigma Aldrich). After 5 days of culture, cells were washed with PBS before fixation in 10% formalin and were stained with Oil Red O (Sigma Aldrich) for 10 minutes.

The article "Isolation and characterization of equine endometrial mesenchymal stromal cells" was published in 2017. Journal: Stem Cell Res Ther.

For osteogenic differentiation, cells were seeded in triplicate wells of 12-well plates (5000 cells/cm^2^) and cultured for 2–4 days before changing medium to DMEM/F-12 containing 10% FBS, 1% penicillin/streptomycin, 10 mM β-glycerophosphate (Sigma Aldrich), 100 nM dexamethasone (Sigma Aldrich), and 200 μM l-ascorbic acid 2-phosphate (Sigma Aldrich). Medium was changed every 2–3 days and after 3 weeks cells were washed with PBS, fixed in 10% formalin, and stained with Alizarin Red (Sigma Aldrich) for 45 minutes.

For chondrogenic differentiation, 3 × 10^5^–4 × 10^5^ cells were centrifuged in a V-bottomed 96-well plate at 720 × *g* for 5 minutes. After centrifugation, without disturbing the freshly formed pellet, medium was changed to DMEM/F-12 containing 1% penicillin/streptomycin, 1% ITS+ premix (Corning), 100 nM dexamethasone (Sigma Aldrich), 200 μM l-ascorbic acid 2-phosphate (Sigma Aldrich), 100 μg/ml sodium pyruvate (Sigma Aldrich), and 10 ng/ml TGF-β1 (R&D Systems). After 24 hours of incubation, the pellets were gently loosened and transferred to a U-bottom 96-well plate with a cell-repellent surface (Greiner bio-one). Micro masses were cultured for 28 days with medium changes every 1–2 days and then fixed in 10% formalin for 24 hours. The pellets were processed and embedded in paraffin. Sections were cut on a microtome (Leica RM2235) and stained with Alcian Blue (Acros Organics) and the nuclear counter stain Nuclear Fast Red (Sigma Aldrich).

### In-vitro smooth muscle differentiation

The protocol used for smooth muscle differentiation was adapted from Guo et al. [31]. In short, endometrial Muc-1^–^ cells and BM MSCs (from three horses each) at passage 3 or 4 were seeded at a density of 70,000 cells/well in triplicate wells of 12-well plates and incubated at 37 °C in 5%CO_2_:95% air for 24 hours before the medium was changed to DMEM containing 1% FBS. After a further 24 hours, differentiation was induced by changing the medium to DMEM containing 1% FBS and 1 ng/ml TGF-β1 (R&D Systems). Control cells were maintained in MSC culture medium and after 7 days all cells were harvested using TRIzol reagent and processed for qPCR analysis as described earlier.

### Statistical analysis

All data were analyzed using IBM SPSS Statistics 22 software using each donor horse as the experimental unit. Normal distribution was tested with the Shapiro–Wilk test and data were log-transformed if necessary. Flow cytometry data were analyzed using Levene’s test for equality of variances and a two-tailed *t* test. QPCR data were analyzed with two-way ANOVA and Tukey’s test. Data are shown as mean ± SEM. Significance was set at *p* < 0.05.

The article "Isolation and characterization of equine endometrial mesenchymal stromal cells" was published in 2017. Journal: Stem Cell Res Ther.

## Results

### Localization of MSC and perivascular markers in equine endometrium

Endometrial tissue was analyzed for the presence of a selection of cluster of differentiation (CD) antigens commonly used to identify human MSCs, namely CD29, CD44, CD90, and CD105 (Fig. 1a), as well as the perivascular cell surface markers, CD146 and NG2 (Fig. 1b). CD29 and CD44 were localized mainly around blood vessels. Milder staining for CD29 was found around endometrial glands and underneath the epithelium. CD90 clone 5E10 was very abundant throughout the stroma, except in glandular cells (data not shown), indicating lack of specificity. CD90 clone OX7 staining was present throughout the endometrial stroma in a string-like pattern, and also around endometrial glands. CD105 staining was less abundant and localized within single cells throughout the stroma. All MSC markers tested were absent from glandular cells and the endometrial epithelium. The perivascular markers, CD146 and NG2, were mostly located around the blood vessel walls.

**Fig. 1:** Immunohistochemistry of equine endometrial sections. Photomicrographs show localization of (**a**) MSC markers CD29, CD44, CD90, and CD105 and (**b**) perivascular markers NG2 and CD146 within the equine endometrium. DAPI was used to stain cell nuclei. *Yellow arrows*, endometrial glands; *white arrows*, blood vessels. *DAPI* 4′,6-diamidine-2′-phenylindole dihydrochloride (Color figure online)

### Isolation and culture of endometrial MSCs

Culture of endometrial tissue directly following collagenase dissociation resulted in epithelial cells adhering quickly to plastic culture ware and eventually outgrowing the stromal cells (Fig. 2a). Thus, we used magnetic beads bound to Muc-1, a surface marker located within the luminal and glandular epithelium (Fig. 2b), to enrich endometrial digests for stromal cells. The resulting Muc-1^–^ fraction, from here onward referred to as endometrial MSCs, was used for culture (Fig. 2c).

**Fig. 2:** Isolation and culture of MSCs. **a** Micrograph showing cells cultured directly following digestion of equine endometrium. Using this procedure, clusters of epithelial cells (*black arrows*) eventually outgrew stromal cells in culture. **b** Section of equine endometrium stained for Mucin-1, showing positive cells in epithelia and glands (*white arrows*). Cell nuclei stained with DAPI. **c** Micrograph of endometrial stromal cells in culture obtained after separation of epithelial cells (shown in **d**) using beads bound to Mucin-1. **e** Cell colonies produced after seeding of endometrial and BM MSCs at low densities. **f** Cloning efficiencies (*CE*) for endometrial MSCs (*n* = 6 horses) and BM MSCs (*n* = 3 horses) at two different seeding densities. *Scale bars*: 1 mm (**a**, **c**–**e**). *BM* bone marrow, *MSC* mesenchymal stromal/stem cell (Color figure online)

Upon initial seeding, endometrial MSCs attached quickly and evenly over the entire culture surface in contrast to BM MSCs which took longer to adhere and tended to grow in clusters. Moreover, doubling times between passages 1 and 2 tended to be shorter for endometrial MSCs than for BM MSCs (2.8 ± 0.6 vs 5.2 ± 1.9 days, respectively, *p* = 0.09). Cloning efficiency (CE) assays performed at passage 2 yielded similar results for both endometrial and BM MSCs, as shown in Fig. 2e, f.

The article "Isolation and characterization of equine endometrial mesenchymal stromal cells" was published in 2017. Journal: Stem Cell Res Ther.

### Expression of MSC and perivascular markers by endometrial MSCs in culture

The expression of MSC and perivascular cell surface markers was analyzed by qPCR and flow cytometry in endometrial and BM MSCs at different passages (Figs. 3 and 4). Moderate differences were detected in transcript levels of MSC markers, including higher overall levels of CD29 and, to a lesser degree, CD105, in endometrial MSCs than in BM MSCs (as indicated in each case by a significant effect of cell type), as well as a slight reduction in overall CD29 levels between passages 1 and 4 (Fig. 3). Flow cytometry (Fig. 4) showed all of these markers to be present, on average, in ≥97% of endometrial and BM MSCs (except for CD105, detected in 80% of BM MSCs). Moreover, there was an overall increase in transcript levels of CD146 between passages 1 and 4 (Fig. 3). The levels of another perivascular marker, NG2, did not change with passage but were lower in endometrial MSCs than in BM MSCs (Fig. 3), a result that was confirmed by flow cytometry data (Fig. 4). Finally, CD34 and MHC-II were expressed by a minority of cells (≤2%) in both endometrial and BM MSC cultures (Fig. 4), whereas CD45 was detectable in BM MSCs at passage 1 only (Fig. 3).

**Fig. 3:** Transcript levels (arbitrary units) of cell surface markers in cultured MSCs. Expression of MSC markers (CD29, CD44, CD90, CD105), perivascular markers (NG2, CD146), and hematopoietic markers (CD34, CD45) quantified by qPCR in endometrial MSCs (*n* = 6 horses, *white bars*) and BM MSCs (*n* = 3 horses, *gray bars*) in culture at passages 1 and 4. All results shown as mean ± SEM. Significant main effects (*p* < 0.05) of passage, cell type, and passage × cell type interaction obtained by two-way ANOVA are shown. *AU* arbitrary units

**Fig. 4:** Flow cytometry analysis. Representative flow cytometry histograms with percentages of endometrial and BM MSCs (*n* = 6 and *n* = 3 horses, respectively) positive for different MSC, perivascular, and hematopoietic cell surface markers. *Grey areas*, signal from isotype controls; *black lines*, signal from the specific cell surface marker. *BM* bone marrow, *MSC* mesenchymal stromal/stem cell

The article "Isolation and characterization of equine endometrial mesenchymal stromal cells" was published in 2017. Journal: Stem Cell Res Ther.

### In-vitro differentiation of endometrial MSCs

The ability of endometrial MSCs to undergo trilineage differentiation was assessed in parallel with that of BM MSCs. Endometrial MSCs differentiated into adipogenic, osteogenic, and, albeit to a lesser degree than BM MSCs, chondrogenic lineages (Fig. 5).

**Fig. 5:** Trilineage differentiation of endometrial MSCs (**a**, **c**, **e**) and BM MSCs (**b**, **d**, **g**). Representative images of endometrial and BM MSCs (*n* = 3 horses each) after differentiation and staining with Oil red O (**a**, **b**), Alizarin Red (**c**, **d**) and Alcian Blue/Nuclear Fast Red (**e**–**g**) to assess differentiation into adipogenic, osteogenic, and chondrogenic lineages, respectively. *Insets* show nondifferentiated control cells (**a**–**d**). Nondifferentiated control BM MSCs used in chondrogenic differentiation experiments shown in (**f**). *Scale bars*: 100 μm (**a**, **b**), 500 μm (**c**, **d**, **e**, **g**) and 1 mm (**f**)

Additionally, the relative capacity of the two types of MSCs to differentiate into smooth muscle, a key component of the myometrium in the uterus, was determined by treating cells with TGF-β1. Endometrial MSCs, but not BM MSCs, underwent morphological changes primarily characterized by shortening of the cell body in response to treatment (Fig. 6a, b). Because of the difficulty of clearly distinguishing smooth muscle cells from undifferentiated MSCs, we assessed the expression of early (ACTA2), intermediate (CNN1), and mature (MYH11) smooth muscle markers [31] in endometrial and BM MSC cultures by qPCR (Fig. 6c). Results showed an increase in mean transcript levels of the intermediate marker, CNN1, in BM MSCs (1.7-fold, *p* < 0.05) and, particularly, in endometrial MSCs (2.9-fold, *p* < 0.0001) between days 0 and 7, and an increase in the levels of the mature smooth muscle marker, MYH11, only in endometrial MSCs (1.8-fold, *p* < 0.005).

**Fig. 6:** Smooth muscle differentiation. Micrographs showing (**a**) endometrial MSCs (*n* = 3 horses) and (**b**) BM MSCs (*n* = 3 horses) induced to differentiate into smooth muscle for 7 days. *Insets* show noninduced control cells. *Scale bars*: 500 μm. **c** Expression of smooth muscle markers in endometrial MSCs (*white bars*) and BM MSCs (*grey b*ars) before (*d0*) and on day 7 (*d7*) of differentiation. Results shown as mean ± SEM. Significant main effects (*p* < 0.05) of day, cell type, and day × cell type interaction obtained by two-way ANOVA are shown. *AU* arbitrary units

The article "Isolation and characterization of equine endometrial mesenchymal stromal cells" was published in 2017. Journal: Stem Cell Res Ther.

## Discussion

MSCs—defined by their adherence to plastic, expression of a subset of cell surface markers, and ability to differentiate into adipogenic, osteogenic, and chondrogenic lineages [3]—have to this date been isolated from several body tissues including bone marrow, fat, umbilical cord, placenta, amniotic fluid, umbilical cord blood, peripheral blood, and endometrium [32–35]. Bone marrow and adipose tissue have been the most common sources of clinical MSCs in horses, and they are also the most common sources used for clinical trials in humans. Collection of MSCs from these locations requires relatively invasive procedures involving sedation and local anesthesia, and carries the potential of postsurgical complications [36]. Thus, alternative sources of equine MSCs, such as the endometrium, are desirable. A major advantage of isolating MSCs from the endometrium compared to bone marrow or adipose tissue is that cells can be harvested by biopsy collection [24, 37], which is a relatively noninvasive approach used routinely in horses for diagnostic purposes that does not require sedation or local anesthesia [38]. In this study, we show for the first time that putative MSCs contained within the equine endometrium can be harvested and expanded in vitro, and have characteristics that may prove useful for tissue regeneration applications.

Endometrial MSCs had typical spindle-shaped morphology, indistinguishable from that of BM MSCs; however, they tended to grow faster than BM MSCs following initial seeding, as indicated by their mean doubling time values. In contrast, cloning efficiencies (CE) at passage 2 were similar for the two cell types, around 25–30%, and comparable to previous reports from 27% [39] to 34% [40] for equine BM MSCs. The faster initial growth of endometrial MSCs relative to BM MSCs may be conferred by their native in-vivo environment characterized by fast tissue turnover during the estrous cycle. If confirmed in future studies, this property of endometrial MSCs may provide an advantage over other MSC sources because it may allow shortening of the interval between collection of tissue samples and transplant of in-vitro expanded MSCs, which is a serious limitation of current BM and adipose MSC treatments in horses. In addition, based on cell yields obtained from 1 g of endometrial tissue (≥10^7^ Muc-1^–^ cells) and considering subsequent growth rates in culture (see Results), we estimate that a typical 0.2–0.4 g biopsy would readily yield >10 million cells after short-term expansion, a sufficient number for therapy applications in horses. Furthermore, when executed appropriately, the biopsy procedure does not result in damage or scarring of the uterus. Indeed, it has been shown that repeated collection of multiple biopsies (up to five each time) before estrus had no effect on subsequent pregnancy rates in mares [41].

The article "Isolation and characterization of equine endometrial mesenchymal stromal cells" was published in 2017. Journal: Stem Cell Res Ther.

Cells staining for CD44, CD105, CD146, and NG2 were located primarily around blood vessels within the equine endometrium, consistent with the identification of perivascular cells as native counterparts of MSCs in many different human tissues [7, 42], including the endometrium [6]. By contrast, CD90 (clone OX7) followed a less restricted pattern throughout the stroma to include nonperivascular cells. The distinct abundance of CD90 compared to the other MSC markers tested suggests that this may not be an appropriate marker for equine MSCs in the endometrium.

Consistent with the definition of MSCs, endometrial stromal cells robustly maintained the expression of CD29, CD44, CD90, and CD105 in culture, as well as, to a lesser extent, perivascular markers, whilst having negligible expression of hematopoietic markers and MHC-II, in agreement with previous studies with human endometrial-derived MSCs [5, 25, 27, 43]. A limited number of studies have compared the features of endometrial MSCs with MSCs from other sources [23, 44]. Our finding based on results of flow cytometry and qPCR, showing that endometrial MSCs in culture display moderately higher levels of CD29, CD90, and CD105 but lower levels of NG2 than their BM counterparts, is consistent with data from Indumathi et al. [23]. Whether this is indicative of differences in the abundance of stem cells between the two tissue sources or reflects tissue-specific changes in immunophenotype that may be induced in culture should be investigated in future studies.

That endometrial and BM MSCs have different properties was confirmed by the results of differentiation assays; specifically by the observation that while endometrial MSCs were able to undergo trilineage differentiation, their ability to generate cartilage was lower than that of BM MSCs based on a clearly reduced intensity of Alcian Blue staining in endometrial MSC-derived chondrogenic pellets (Fig. 5). In contrast, the opposite was observed in relation to the ability of MSCs to adopt a smooth muscle phenotype, as evidenced by a distinct increase in endometrial MSCs, but not in BM MSCs, in the levels of the mature smooth muscle marker, MYH11, after treatment with TGF-β1. There is evidence that significant differentiation bias can be conferred by the tissue of origin of MSCs [45]. For example, while human multipotent cell populations from the myometrium and skeletal muscle had a similar immunophenotype and ability to differentiate into smooth muscle, only skeletal muscle-derived progenitors were able to undergo osteogenic and adipogenic differentiation [46]. In light of this, a distinct ability of endometrial MSCs (compared to BM MSCs) to differentiate into smooth muscle may be related to the presence of a large smooth muscle component in the uterus, the myometrium. Whether our observation alternatively reflects the presence, natural or through contamination during sample collection, of myometrial precursor cells, different from MSCs, in the endometrial stroma needs to be investigated in future studies. Nonetheless, a reported intrinsic ability of human endometrial MSCs to differentiate into smooth muscle provides the rationale for specific therapeutic applications already being sought for these cells (e.g., pelvic organ prolapse) [47].

The article "Isolation and characterization of equine endometrial mesenchymal stromal cells" was published in 2017. Journal: Stem Cell Res Ther.

## Conclusion

We report for the first time the identification, culture, and characterization of stromal cells within the equine uterus that fulfill the definition of MSCs based on clonogenicity, immunophenotype, and ability to differentiate into different mesenchymal derivatives. Although not addressed in this study, the relative abundance and phenotype of MSCs in the equine endometrium may vary with the reproductive stage, a possibility that should be investigated in the future. Endometrial MSCs may provide an easily accessible alternative to therapeutic applications that currently use bone marrow and adipose MSCs in the horse. They may moreover provide a new therapeutic venue for equine uterine disease, a multifaceted and highly prevalent condition which significantly impairs fertility in mares. With this in mind, future studies should be aimed at exploring the clinical regenerative potential of these cells in the endometrium but also in other tissues that have been more commonly targeted with cell therapies, such as musculoskeletal tissue.

## Abbreviations

BM: Bone marrow
BSA: Bovine serum albumin
CD: Cluster of differentiation
CE: Cloning efficiency
DAPI: 4′,6-Diamidine-2′-phenylindole dihydrochloride
EDTA: Ethylenediaminetetraacetic acid
FBS: Fetal bovine serum
MSC: Mesenchymal stromal/stem cell
PBS: Phosphate buffered saline
qPCR: Quantitative polymerase chain reaction

## References

[1] Thomas ED, Lochte HL, Lu WC, Ferrebee JW (1957). Intravenous infusion of bone marrow in patients receiving radiation and chemotherapy. N Engl J Med.

The article "Isolation and characterization of equine endometrial mesenchymal stromal cells" was published in 2017. Journal: Stem Cell Res Ther.

[2] Friedenstein AJ, Piatetzky S, Petrakova KV (1966). Osteogenesis in transplants of bone marrow cells. J Embryol Exp Morphol.

[3] Dominici M, Le Blanc K, Mueller I, Slaper-Cortenbach I, Marini F, Krause D (2006). Minimal criteria for defining multipotent mesenchymal stromal cells. The International Society for Cellular Therapy position statement. Cytotherapy.

[4] Bourin P, Bunnell BA, Casteilla L, Dominici M, Katz AJ, March KL (2013). Stromal cells from the adipose tissue-derived stromal vascular fraction and culture expanded adipose tissue-derived stromal/stem cells: a joint statement of the International Federation for Adipose Therapeutics and Science (IFATS) and the International Society for Cellular Therapy (ISCT). Cytotherapy.

[5] Gargett CE, Schwab KE, Zillwood RM, Nguyen HPT, Wu D (2009). Isolation and culture of epithelial progenitors and mesenchymal stem cells from human endometrium. Biol Reprod.

[6] Schwab KE, Gargett CE (2007). Co-expression of two perivascular cell markers isolates mesenchymal stem-like cells from human endometrium. Hum Reprod.

[7] Crisan M, Yap S, Casteilla L, Chen CW, Corselli M, Park TS (2008). A perivascular origin for mesenchymal stem cells in multiple human organs. Cell Stem Cell.

[8] Caplan AI (2016). MSCs: the sentinel and safe-guards of injury. J Cell Physiol.

[9] Trounson A, McDonald C (2015). Stem cell therapies in clinical trials: progress and challenges. Cell Stem Cell.

[10] Ranera B, Lyahyai J, Romero A, Vazquez FJ, Remacha AR, Bernal ML (2011). Immunophenotype and gene expression profiles of cell surface markers of mesenchymal stem cells derived from equine bone marrow and adipose tissue. Vet Immunol Immunopathol.

[11] Radcliffe CH, Flaminio MJ, Fortier LA (2010). Temporal analysis of equine bone marrow aspirate during establishment of putative mesenchymal progenitor cell populations. Stem Cells Dev.

[12] Godwin EE, Young NJ, Dudhia J, Beamish IC, Smith RK (2012). Implantation of bone marrow-derived mesenchymal stem cells demonstrates improved outcome in horses with overstrain injury of the superficial digital flexor tendon. Equine Vet J.

[13] Smith RK, Korda M, Blunn GW, Goodship AE (2003). Isolation and implantation of autologous equine mesenchymal stem cells from bone marrow into the superficial digital flexor tendon as a potential novel treatment. Equine Vet J.

[14] Lovati AB, Corradetti B, Lange Consiglio A, Recordati C, Bonacina E, Bizzaro D (2011). Comparison of equine bone marrow-, umbilical cord matrix and amniotic fluid-derived progenitor cells. Vet Res Commun.

[15] Reed SA, Johnson SE (2008). Equine umbilical cord blood contains a population of stem cells that express Oct4 and differentiate into mesodermal and endodermal cell types. J Cell Physiol.

The article "Isolation and characterization of equine endometrial mesenchymal stromal cells" was published in 2017. Journal: Stem Cell Res Ther.

[16] Hoynowski SM, Fry MM, Gardner BM, Leming MT, Tucker JR, Black L (2007). Characterization and differentiation of equine umbilical cord-derived matrix cells. Biochem Biophys Res Commun.

[17] Mohanty N, Gulati BR, Kumar R, Gera S, Kumar P, Somasundaram RK (2014). Immunophenotypic characterization and tenogenic differentiation of mesenchymal stromal cells isolated from equine umbilical cord blood. In Vitro Cell Dev Biol Anim.

[18] Letouzey V, Tan KS, Deane JA, Ulrich D, Gurung S, Ong YR, et al. Isolation and characterisation of mesenchymal stem/stromal cells in the ovine endometrium. PLoS One. 2015;10(5):e0127531.10.1371/journal.pone.0127531PMC443636325992577

[19] Miernik K, Karasinski J (2012). Porcine uterus contains a population of mesenchymal stem cells. Reproduction.

[20] Chan RWS, Schwab KE, Gargett CE (2004). Clonogenicity of human endometrial epithelial and stromal cellss. Biol Reprod.

[21] Chan RW, Gargett CE (2006). Identification of label-retaining cells in mouse endometrium. Stem Cells.

[22] De Cesaris V, Grolli S, Bresciani C, Conti V, Basini G, Parmigiani E, et al. Isolation, proliferation and characterization of endometrial canine stem cells. Reprod Domest Anim. 2017;52(2):235–42.10.1111/rda.1288527925313

[23] Indumathi S, Harikrishnan R, Rajkumar JS, Sudarsanam D, Dhanasekaran M (2013). Prospective biomarkers of stem cells of human endometrium and fallopian tube compared with bone marrow. Cell Tissue Res.

[24] Schuring AN, Schulte N, Kelsch R, Ropke A, Kiesel L, Gotte M (2011). Characterization of endometrial mesenchymal stem-like cells obtained by endometrial biopsy during routine diagnostics. Fertil Steril.

[25] Gaafar T, Hawary RE, Osman A, Attia W, Hamza H, Brockmeier K (2014). Comparative characteristics of amniotic membrane, endometrium and ovarian derived mesenchymal stem cells: a role for amniotic membrane in stem cell therapy. Middle East Fertil Soc J.

[26] Wolff EF, Gao XB, Yao KV, Andrews ZB, Du H, Elsworth JD (2011). Endometrial stem cell transplantation restores dopamine production in a Parkinson's disease model. J Cell Mol Med.

[27] Lai D, Wang F, Yao X, Zhang Q, Wu X, Xiang C (2015). Human endometrial mesenchymal stem cells restore ovarian function through improving the renewal of germline stem cells in a mouse model of premature ovarian failure. J Transl Med.

[28] Emmerson SJ, Gargett CE (2016). Endometrial mesenchymal stem cells as a cell based therapy for pelvic organ prolapse. World J Stem Cells.

[29] Aupperle H, Ozgen SHA, Schoon D, Hoppen HO, Sieme H, Tannapfel A (2000). Cyclical endometrial steroid hormone receptor expression and proliferation intensity in the mare. Equine Vet J.

The article "Isolation and characterization of equine endometrial mesenchymal stromal cells" was published in 2017. Journal: Stem Cell Res Ther.

[30] RefFinder. http://leonxie.esy.es/RefFinder/. Accessed 15 July 2016.

[31] Guo X, Stice SL, Boyd NL, Chen SY (2013). A novel in vitro model system for smooth muscle differentiation from human embryonic stem cell-derived mesenchymal cells. Am J Physiol Cell Physiol.

[32] Erices A, Conget P, Minguell JJ (2000). Mesenchymal progenitor cells in human umbilical cord blood. Br J Haematol.

[33] Busser H, Najar M, Raicevic G, Pieters K, Velez Pombo R, Philippart P (2015). Isolation and characterization of human mesenchymal stromal cell subpopulations: comparison of bone marrow and adipose tissue. Stem Cells Dev.

[34] Chang CJ, Yen ML, Chen YC, Chien CC, Huang HI, Bai CH (2006). Placenta-derived multipotent cells exhibit immunosuppressive properties that are enhanced in the presence of interferon-gamma. Stem Cells.

[35] Kim J, Lee Y, Kim H, Hwang KJ, Kwon HC, Kim SK (2007). Human amniotic fluid-derived stem cells have characteristics of multipotent stem cells. Cell Prolif.

[36] Durando MM, Zarucco L, Schaer TP, Ross M, Reef VB (2006). Pneumopericardium in a horse secondary to sternal bone marrow aspiration. Equine Vet Educ.

[37] Revel A (2009). Multitasking human endometrium: a review of endometrial biopsy as a diagnostic tool, therapeutic applications, and a source of adult stem cells. Obstet Gynecol Surv.

[38] Snider TA, Sepoy C, Holyoak GR (2011). Equine endometrial biopsy reviewed: observation, interpretation, and application of histopathologic data. Theriogenology.

[39] Arnhold SJ, Goletz I, Klein H, Stumpf G, Beluche LA, Rohde C (2007). Isolation and characterization of bone marrow-derived equine mesenchymal stem cells. Am J Vet Res.

[40] Bourzac C, Smith LC, Vincent P, Beauchamp G, Lavoie JP, Laverty S (2010). Isolation of equine bone marrow-derived mesenchymal stem cells: a comparison between three protocols. Equine Vet J.

[41] Watson ED, Sertich PL (1992). Effect of repeated collection of multiple endometrial biopsy specimens on subsequent pregnancy in mares. J Am Vet Med Assoc.

[42] da Silva ML, de Deus Wagatsuma VM, Malta TM, Bonini Palma PV, Araujo AG, Panepucci RA, et al. The gene expression profile of non-cultured, highly purified human adipose tissue pericytes: transcriptomic evidence that pericytes are stem cells in human adipose tissue. Exp Cell Res. 2016;349(2):239–54.10.1016/j.yexcr.2016.10.01727789253

[43] Dimitrov R, Timeva T, Kyurkchiev D, Stamenova M, Shterev A, Kostova P (2008). Characterization of clonogenic stromal cells isolated from human endometrium. Reproduction.

[44] Gaafar T, Osman O, Osman A, Attia W, Hamza H, El Hawary R (2014). Gene expression profiling of endometrium versus bone marrow-derived mesenchymal stem cells: upregulation of cytokine genes. Mol Cell Biochem.

The article "Isolation and characterization of equine endometrial mesenchymal stromal cells" was published in 2017. Journal: Stem Cell Res Ther.

[45] Sacchetti B, Funari A, Remoli C, Giannicola G, Kogler G, Liedtke S (2016). No identical “mesenchymal stem cells” at different times and sites: human committed progenitors of distinct origin and differentiation potential are incorporated as adventitial cells in microvessels. Stem Cell Reports.

[46] Pierantozzi E, Vezzani B, Badin M, Curina C, Severi FM, Petraglia F (2016). Tissue-specific cultured human pericytes: perivascular cells from smooth muscle tissue have restricted mesodermal differentiation ability. Stem Cells Dev.

[47] Gargett CE, Schwab KE, Deane JA (2016). Endometrial stem/progenitor cells: the first 10 years. Hum Reprod Update.

